# Investigating Pollen and Gene Flow of WYMV-Resistant Transgenic Wheat N12-1 Using a Dwarf Male-Sterile Line as the Pollen Receptor

This article has been retracted.

**DOI:** 10.1371/journal.pone.0151373

**Published:** 2016-03-14

**Authors:** Shanshan Dong, Yan Liu, Cigang Yu, Zhenhua Zhang, Ming Chen, Changyong Wang

**Affiliations:** 1 Nanjing Institute of Environmental Sciences, Ministry of Environmental Protection, Nanjing, China; 2 Key Laboratory on Biosafety of Environmental Protection, Ministry of Environmental Protection, Nanjing, China; 3 Key Laboratory of Biology and Genetic Improvement of Triticeae Crops, Institute of Crop Sciences, Chinese Academy of Agricultural Sciences, Beijing, China; Huazhong University of Science and Technology, CHINA

## Abstract

Pollen-mediated gene flow (PMGF) is the main mode of transgene flow in flowering plants. The study of pollen and gene flow of transgenic wheat can help to establish the corresponding strategy for preventing transgene escape and contamination between compatible genotypes in wheat. To investigate the pollen dispersal and gene flow frequency in various directions and distances around the pollen source and detect the association between frequency of transgene flow and pollen density from transgenic wheat, a concentric circle design was adopted to conduct a field experiment using transgenic wheat with resistance to wheat yellow mosaic virus (WYMV) as the pollen donor and dwarf male-sterile wheat as the pollen receptor. The results showed that the pollen and gene flow of transgenic wheat varied significantly among the different compass sectors. A higher pollen density and gene flow frequency was observed in the downwind SW and W sectors, with average frequencies of transgene flow of 26.37 and 23.69% respectively. The pollen and gene flow of transgenic wheat declined dramatically with increasing distance from its source. Most of the pollen grains concentrated within 5 m and only a few pollen grains were detected beyond 30 m. The percentage of transgene flow was the highest where adjacent to the pollen source, with an average of 48.24% for all eight compass directions at 0 m distance. Transgene flow was reduced to 50% and 95% between 1.61 to 3.15 m, and 10.71 to 20.93 m, respectively. Our results suggest that climate conditions, especially wind direction, may significantly affect pollen dispersal and gene flow of wheat. The isolation-by-distance model is one of the most effective methods for achieving stringent transgene confinement in wheat. The frequency of transgene flow is directly correlated with the relative density of GM pollen grains in air currents, and pollen competition may be a major factor influencing transgene flow.

## Introduction

Crop-to-crop gene flow in agricultural production is a universal occurrence and is a principal factor affecting the varietal purity of cultivated crops [1]. In recent years, with the spread and increasing growing area of genetically modified (GM) crops on a global scale, how best to control the escape of an exogenous gene from GM crops to non-GM crops has aroused great biosafety concerns [2–5]. Transgenes conferring novel traits with a strong selective advantage escaping into conventional crops or wild relatives through gene flow could result in regional or international trade disputes in seed markets or potential ecological consequences. Thus, a field study of transgene flow from GM crop to non-GM crop is an essential first step for a complete evaluation of gene flow and its potential consequences, which will provide a solid base for environmental risk assessment.

Transgene flow can occur by pollen dispersal or by direct movement of seed or vegetative propagules [6]. Pollen-mediated gene flow (PMGF) is the main mode of transgene flow in flowering plants because pollen is the important vehicle for disseminating transferred alien genes [7]. The study of pollen flow is a necessary component in the ecological risk assessment of transgene escape. Previous studies have shown that the pollen flows of different plants differed significantly in their dispersal patterns and that there might be different models for the same plants under various environment and weather conditions [8–12]. Especially in wind-pollinated plants, pollen dispersal can be greatly affected by pollen grain architecture, pollen shape and climatic factors (e.g. weather conditions during blooming period, wind speed and direction, day and night temperature, light and relative air humidity) [13,14]. It is therefore vital to investigate in detail the mode of pollen dissemination for a particular species under field conditions.

Wheat (*Triticum aestivum L*.) is a wind-pollinated and predominantly self-pollinating crop. The frequency of PMGF in common wheat cultivars is usually low, and the average cross-pollination rate is 1–2% for plants in close proximity [15–17]. However, outcrossing rates may be very different in various trials due to geographic location, wheat genotypes used, experimental approach and environmental conditions directly related to the amount of wind-borne pollen [18, 19]. By using two GM spring wheat lines as pollen donors, Foetzki et al. (2012) detected 185,000 seedlings from seeds collected around the experimental field up to a distance of 200 m, and found only three outcrosses in the border crop surrounding the pollen source [20]. Loureiro et al. (2007) used emasculated wheat as pollen receptor to conduct a 3-year study and assessed the maximum potential outcrossing between two wheat cultivars (*Triticum aestivum* L.) and between wheat and durum wheat (*Triticum turgidum* L. var. *durum*), the result showed that cross-pollination at 0 m distance ranged from 37 to 56% for *T*. *aestivum* cultivars and 5 to 30% with *T*. *turgidum* in the absence of any pollen competition [21]. In further studies, Loureiro et al. (2012) investigated the frequency of PMGF in transgenic wheat at two locations using three conventional wheat species, and found that a maximum outcrossing rate of 3.5% near the pollen source, averaging 0.029% and 0.337% at 0 m distance, respectively [22]. Although the gene flow of wheat generally occurs at extremely low frequencies and over very short distances, effective measures should be taken to control the contamination of adjacent non-transgenic wheat crops.

At present, there are no commercial GM wheat varieties but a number of transgenic wheat lines have been successfully developed and field-tested, and there are extensive researches on a wide range of GM wheat traits, such as herbicide tolerance, virus resistance and drought resistance [23–25]. There is concern that once transgenic wheat is released for commercial production, there is potential for pollen flow from GM wheat to non GM-wheat. One of the most effective methods for preventing outcrossing and contamination between compatible genotypes is the use of isolation distances [26]. A field study was conducted in western Canada to measure the PMGF from a 16-ha (400 × 400 m) field of imidazolinone (IMI)-resistant wheat to an adjacent field of conventional wheat and found the observed maximum PMGF was 0.2% at the common border (0.5 m distance) but declined exponentially with increasing distance from pollen source: by more than 50% at a 5 m distance from the pollen donor [27]. Rieben et al. (2011) reported that the cross-pollination rate varied among the eight wheat lines tested from 0.5–8.5%, with an average of 3.36% within a GM wheat field, and that outcrossing declined from 0.7 to 0.03% over the test distances of 0.5 to 2.5 m from pollen donors [28]. A study carried out by Matus-Cádiz et al. (2007) indicated that gene flow in wheat occurs at trace levels (≤0.01%) at distances up to 2.75 km [12]. These studies suggested that the PMGF frequency varies widely between experiments for a same set of isolation distances due to environmental conditions, which have a large influence on pollen dispersal [29]. In addition, the distribution of pollen grains is closely related to genetic background of pollen donor which determines the pollen grain architecture and shape, pollen flow patterns may differ depending on the genotype of transgenic wheat varieties. Thus, further studies on pollen and gene flow of transgenic wheat are needed prior to the release and commercialization of any specific transgenic cultivars, which can help to establish isolation distances to enable the coexistence of conventional wheat varieties with GM wheat.

Wheat yellow mosaic disease (WYMV) has caused serious yield losses in the major wheat-growing areas in China, which is characterized by mosaic or yellow-striped leaves and plant stunting [30, 31]. Transgenic wheat with durable and broad-spectrum resistance to WYMV will alleviate the damage caused by WYMV [32]. In this study we used GM lines of winter wheat with transgenes conferring resistance against WYMV as pollen donor to assess pollen and gene flow by adopting a concentric circle design. In order to enhance detection sensitivity and differentiate gene flow frequency in the various compass directions, dwarf male-sterile wheat (hereafter: DMSW) with a higher outcrossing rate was used as pollen receptor. Owing to the heterozygous male sterile gene, the DMSW pollinated with non-dwarf varieties always gives rise to half dwarf sterile progeny and half non-dwarf fertile progeny. Therefore, there were 50% non-dwarfing fertile plants in the DMSW populations in this study.

The objectives of this study were to: (1) detect the patterns of pollen dispersal and gene flow frequency in various directions around the pollen source; (2) measure the influence of the distance between the GM pollen donor and the non-GM pollen recipient on the pollen and gene flow; (3) test for the association of transgene flow frequency with the pollen density from transgenic wheat.

## Materials and Methods

### Materials

In this study, the marker-free WYMV-resistant transgenic winter wheat line N12-1 containing an antisense *NIb8* gene (the NIb replicase of WYMV) served as a pollen donor. The line was generated by the Institute of Crop Science, Chinese Academy of Agricultural Sciences, and has previously been described by Chen et al. [32]. Briefly, the vector pubi-NIb containing the *NIb8* gene and the assistant plasmid pAHC20 with the *bar* selectable marker gene were first co-transformed into wheat variety Yangmai 158 by particle bombardment, resulting in the four transgenic lines (N12, N13, N14 and N15). Transgenic wheat lines were shown to be homozygous in the *Nib8* insertion locus after the T3 generation by PCR. The marker-free transgenic wheat line N12-1 was obtained by PCR and herbicide resistance testing of the T3 plants derived from the positive N12 line. The transgenic wheat line received permission from the National Biosafety Committee of China for pre-release production tests under controlled field conditions. Dwarf male-sterile wheat used as a receiver of transgenic pollen was a Taigu genic male sterile (no seed setting by self-pollination) wheat with dwarf marker, which was provided by the Xuzhou Academy of Agricultural Sciences, Jiangsu Province, China.

### Field experimental design

The experiment was conducted from October 2011 until June 2012 at an experimental area with restricted access in Xuzhou Academy of Agricultural Sciences, Jiangsu Province, China. This area was approved by the National Biosafety Committee of China for growing transgenic wheat for environmental biosafety assessments. A diagrammatic presentation of the experimental design is shown in Fig 1. The pollen donor plot was designed as a circular area of 78.5 m^2^ with a radius of 5 m and located at the center of the field (Fig 1). The concentric circle of the recipient was equally divided into eight compass sectors (N, NE, E, SE, S, SW, W, NW) with a radius of 50 m and the recipient DMSW plants were planted in each sector (Fig 1). Wheat was seeded by direct drill in rows 20 cm apart. We adjusted the sowing date of the donor and recipient in order to synchronize their flowering times. N12-1 seeds were sown on 20th October and DMSW seeds were sown on 10th November. Management of the experimental materials and cultivation practices followed the usual procedures by local farmers. No pesticides were applied to the field.

**Fig 1:** Diagrammatic presentation of the experimental design. The circular pollen donor N12-1 plot with radius 5m was planted at the center of experiment field. Pollen recipient dwarf male-sterile wheat (DMSW) was grown at eight compass directions. The radius of concentric circle of the recipient DMSW was 50 m.

### Pollen flow measurement

Winter wheat’s flowering time is generally from late-April to early-May, with the peak hours being from 9:30 to 12:00 A.M. each day. We recorded the pollen flow in eight different directions around the pollen donor plot during the peak flowering period of transgenic wheat between the 27th and 29th April 2012. To reduce the impact of pollen grains from non-dwarfing fertile plants in the recipient groups in the process of detecting pollen flow, we removed the non-dwarfing plants that were mixed with the dwarfing sterile plants by hand at booting stage. The circumference of the pollen donor was used as a starting point and the pollen flow of each direction was measured at distance intervals of 0, 1, 2, 3, 5, 10, 20 and 50 m. Pollen density was measured using the pollen trap method described by Song et al. [7]. Five microscope glass slides (7.6 × 2.6 cm^2^) were coated with vaseline and placed on a 45 cm high stool close to the DMSW flower height level. On sunny days, microscope slides were set up at ~8:30 A.M. before flowering and collected around 3:30 P.M., after most flowers had discharged. The collected smears of glass slides were observed under a microscope after staining with aniline blue in lacto phenol. The number of pollen grains was counted and the pollen density calculated as the number of grains per cm^2^. During the wheat flowering period, the atmospheric parameters, including temperature, air humidity, wind speed, and wind direction near the experimental field were recorded each hour, which were provided by the Xuzhou National Basic Weather Stations.

### Seed set measurement

At seed maturity, seeds from the DMSW were hand harvested at distance intervals of 0, 1, 2, 3, 5, 10, 20 and 50 m from the pollen source in each compass sector. Each sampling zone was equally divided into three segments (as three replicates) and the seeds from the recipient plants at different distances in each replicate were individually harvested. We harvested about 50 wheat spikes at each sample zone, and assessed the seed set per spike by calculating the proportion of the total number of seeds produced per spike to total number of florets per spike. Finally, all harvested seeds from each replicate at each sample zone were mixed and were germinated for the identification of transgenic hybrids.

### Detection of transgene flow

The sampled seeds were germinated at 28°C in a light growth chamber. Leaf samples were collected from individuals for DNA extraction approximately 15 d after seed germination. Genomic DNA was extracted using the GMO Crop Extraction & Amplification Kit (KG202 TIANGEN). PCR analysis of the target transgenic *NIb8* gene was conducted using the primer pair: NIb8F 5′-GCGACAAACCTGAAAGCCCCACAC-3′; NIb8R 5′-AACGCCGCCCTTCTTAGCCCACT-3′. The PCR-amplified fragment was expected to be 593 bp (Fig 2). The total volume of the PCR was 20 μL, containing 1.0 μL of buffer (mix), 0.6 μL of primers (10 pM), 0.6 μL of template, 0.4 μL of Taq polymerase (5 U/μL) and 7.8 μL of double-distilled H_2_O. The amplification conditions were 94°C for 5 min for denaturing; 94°C for 30 s, 65°C for 30 s, 72°C for 30 s, for 35 cycles for amplification; and 72°C for 10 min for elongation. The PCR products were detected by electrophoresis using 1% agarose-ethidium bromide gels. The frequency of transgene flow at different distances in each compass sector was determined as the ratio of number of transgenic seedlings against the total number of seedlings examined.

**Fig 2:** PCR detection of the *NIb8* gene in dwarf male-sterile wheat (DMSW) seeding. M, DNA marker; lane1, positive control (N12-1); lanes 2–5, genetically modified (GM) seedling with the *NIb8* gene; lanes 6–8, nongenetically modified (non-GM) seedling; lane 9, negative control (H_2_O).

### Data analysis

A one-way ANOVA procedure was performed to detect statistical differences in pollen density, seed set and transgene flow frequency among the various directions. Student–Newman–Keuls (SNK) multiple comparisons tests were used to compare the level of statistical significance and a P value of <0.05 was taken as the level for significance. In order to estimate the pollen and transgene flow in relation to the distance from the pollen source, the exponential decay model for each sector was fitted to the data: y = a ∙ exp^(−bx)^, where y represents pollen density (grain/cm^2^) or transgene flow frequency (%); x represents the distance (m) from the pollen source; a is the intercept and b is the curve parameter determining the slope of the curve (decline rate). The distances wherein transgene flow frequency was reduced by 50 and 95% (o_50_ and o_95_) were estimated from the exponential decay function following the equations [33]:

$$o_{50}=\frac{\ln(0.5\times a)-\ln\;a}{-b}$$

$$o_{95}=\frac{\ln(0.01\times a)-\ln\;a}{-b}$$

In addition, the association between the pollen density and gene flow frequency was determined using a linear regression model. All statistical analyses were performed using SPSS19.0.

## Results

### Pollen flow of transgenic wheat in the eight compass sectors

ANOVA analysis revealed significant differences in pollen dispersal among the eight compass sectors at distances of 0–20 m from the pollen donor. When the distance increased up to 30 m, no significant difference was observed among geographical orientations (Table 1). More pollen grains were observed in the SW, W, NW, SE and S sectors that were downstream of the prevailing or sub-dominant wind and the highest pollen density appeared in the SW sector (Table 1). Less pollen grains were observed in the NE, E, and N sectors that were lateral to or upstream of the prevailing wind direction and the lowest pollen density appeared in the NE sector (Table 1).

**Table 1:** One-way ANOVA for the pollen density detected in different compass sectors.

Distances(m)	Pollen density in eight compass sectors							
	E	SE	S	SW	W	NW	N	NE
0	201.07±4.02^d^	399.65±5.77^b^	297.24±2.89^c^	487.07±6.26^a^	407.14±4.93^b^	345.95±9.01^c^	203.57±5.6^d^	118.65±4.7^e^
1	51.21±3.04^e^	102.41±4.53^c^	111.15±3.68^c^	198.58±4.72^a^	157.36±3.68^b^	114.9±3.6^c^	73.69±4.67^d^	43.71±3.42^e^
2	26.23±3.2^d^	27.48±2.67^d^	64.94±3.6^c^	126.14±4.29^a^	96.17±3.7^b^	44.96±6.46^cd^	36.22±4.35^cd^	32.47±2.62^cd^
5	7.49±2.29^b^	5±3.34^b^	24.98±4.6^ab^	39.97±2.67^a^	23.73±3.2^ab^	22.48±4.11^ab^	5±2.29^b^	13.74±2.85^b^
10	5±1.67^b^	3.75±2.36^b^	24.98±3.64^a^	27.48±2.67^a^	1.25±1.67^b^	5±2.29^b^	3.75±2.89^b^	7.49±2.29^b^
20	1.25±1.67^b^	1.25±1.67^b^	2.5±2.36^b^	21.23±2.36^a^	1.25±1.67^b^	2.5±2.36^b^	2.5±1.85^b^	2.5±1.85^b^
30	0	1.25±1.67	1.25±1.67	1.25±1.67	0	0	3.75±2.89	1.25±1.67
50	0	1.25±1.67	1.25±1.67	0	0	0	0	0

Data are expressed as the mean number of pollen grains at each distance and numbers in parentheses indicate the standard errors of the means. Different letters following the average values denote their significant differences (*P* < 0.05) under statistical analysis using the Student–Newman–Keuls (SNK) test.

Regression analysis indicated that pollen dispersal dramatically reduced in all orientations with increasing distance (Table 2). Most of the pollen grains were concentrated within 5 m from the pollen source and only a few pollen grains were detected at >30 m. However, the descending rate of pollen flow in various orientations was significantly different. The exponential decay models for each direction revealed the decline speed in the higher pollen density sectors (SW and W) was relatively slow compared to that in the lower pollen density sectors (E and NE) (Table 2). The results demonstrated that weather conditions, especially wind direction, had a strong influence on the descending rate of pollen dispersal.

**Table 2:** The exponential decay models for pollen and gene flow of transgenic wheat and the corresponding determination coefficient (R^2^) in eight compass sectors.

Directions	pollen flow		gene flow	
	y = a ∙ exp^(−bx)^	R^2^	y = a ∙ exp^(−bx)^	R^2^
E	y = 200.21 ∙ exp^(−1.25x)^	0.994	y = 31.93 ∙ exp^(−0.43x)^	0.851
SE	y = 399.57 ∙ exp^(−1.36x)^	0.999	y = 54.73 ∙ exp^(−0.43x)^	0.937
S	y = 293.89 ∙ exp^(−0.86x)^	0.980	y = 48.45 ∙ exp^(−0.26x)^	0.953
SW	y = 479.79 ∙ exp^(−0.76x)^	0.983	y = 69.05 ∙ exp^(−0.22x)^	0.968
W	y = 402.45 ∙ exp^(−0.82x)^	0.993	y = 62.65 ∙ exp^(−0.23x)^	0.961
NW	y = 345.08 ∙ exp^(−1.06x)^	0.995	y = 48.95 ∙ exp^(−0.35x)^	0.92
N	y = 202.59 ∙ exp^(−0.95x)^	0.997	y = 31.73 ∙ exp^(−0.28x)^	0.916
NE	y = 116.02 ∙ exp^(−0.77x)^	0.969	y = 21.49 ∙ exp^(−0.33x)^	0.927

### Seed set of dwarf male-sterile wheat among different geographical orientations

There was significant variance in seed set of DMSW among different geographical orientations (Table 3). Statistical analysis showed that the DMSW at downwind sectors (SW, W and S) had a relatively higher seed set, with average seed sets of 13.70, 12.03 and 10.52% respectively. The DMSW at upwind sectors (NW, SE and NE), by contrast, had lower seed sets, with average seed sets of less than 7%, suggesting that the pollen dispersal from pollen donor had an obvious effect on the seed set of pollen receptor DMSW. The seed set of DMSW in all orientations declined rapidly as the distance from the pollen source increased, and the average seed set had been reduced to less than 10% at 3 m from the edge of pollen donor. However, it was found that the changing patterns of the seed set were different among the various orientations, which were similar to the pollen dispersal modes of the pollen donor.

**Table 3:** One-way ANOVA for the seed set of dwarf male-sterile wheat (DMSW) in different compass sectors.

Distances(m)	Seed set in eight compass sectors (%)								
	E	SE	S	SW	W	NW	N	NE	P
0	20.75±3.13^bcd^	11.98±2.01^cd^	22.15±2.66^abc^	31.75±3.56^a^	25.20±3.74^ab^	12.49±3.07^cd^	9.52±1.43^d^	14.87±3.54^bcd^	0.000***
1	19.61±3.33^a^	14.80±2.50^ab^	13.81±2.02^ab^	16.90±2.31^ab^	19.20±3.17^a^	11.41±2.12^ab^	6.41±2.07^b^	13.03±2.86^ab^	0.025*
2	5.84±1.39^b^	7.49±1.91^b^	9.31±1.56^b^	16.30±2.61^a^	12.58±2.19^ab^	8.79±2.20^b^	6.72±1.52^b^	5.03±1.40^b^	0.000***
5	3.30±1.06^c^	8.50±2.39^abc^	8.74±1.41^abc^	12.56±1.92^ab^	14.25±2.97^a^	7.42±1.66^abc^	12.21±1.79^ab^	5.75±1.03^bc^	0.000***
10	2.36±0.78^d^	3.14±0.93^cd^	9.47±2.02^b^	15.11±2.79^a^	8.23±1.61^bc^	2.72±0.68^cd^	8.44±1.55^bc^	3.79±0.88^cd^	0.000***
20	2.45±0.75	7.21±2.34	7.92±1.44	8.06±1.39	5.71±0.79	3.42±0.80	6.66±1.72	6.24±1.05	0.072NS
30	5.94±1.77^b^	1.65±0.50^b^	9.54±1.68^a^	5.06±1.20^b^	4.79±0.67^b^	4.84±0.98^b^	3.86±1.19^b^	4.58±1.06^b^	0.007**
50	3.43±1.14^ab^	2.60±0.64^ab^	3.22±0.68^ab^	3.83±1.39^ab^	6.25±1.53^a^	0.52±0.28^b^	6.61±0.88^a^	4.72±1.72^ab^	0.002**

Data are expressed as the mean value of seed set at each distance and numbers in parentheses indicate the standard errors of the means. Different letters following the average values denote their significant differences (*P* < 0.05) under statistical analysis using the Student–Newman–Keuls (SNK) test. NS, not significant.

*P < 0.05

**P < 0.01

***P < 0.001.

### Frequency of transgene flow to DMSW in the eight compass sectors

The flowering period of wheat was from late-April to early-May in 2012. The flowering time of the pollen donor transgenic wheat was matched to that of the recipient DMSW by adjusting the sowing date in the experiment. A total of 6,799 seeds from over 3,200 DMSW spikes were collected and germinated in eight compass sectors. The average germination rate was 72.8%, and 4,952 seeding were examined by PCR analysis of the target transgenic *NIb8* gene. Analysis of transgene flow frequency in the different directions revealed that there were significant differences among the eight compass sectors within 5 m from the pollen source, while no significant statistical difference was detected over 10 m (Table 4). A clearly higher transgene flow frequency was observed in the downwind SW and W sectors, with average frequencies from 0 to 50 m being 26.37 and 23.69%, respectively. A relatively low frequency was observed in the upwind NE, N and E sectors and the average cumulative frequencies from 0 to 50 m were 7.02, 9.87 and 10.88%, respectively. Our data suggest that wind direction plays a significant role in the pattern of wheat gene flow, which matched the pollen flow examined during the flowering period. The frequency of transgene flow is closely related to pollen density from transgenic wheat (R^2^ = 0.857, P<0.001).

**Table 4:** One-way ANOVA for the transgene flow frequency in different compass sectors.

Distances(m)	Transgene flow frequencies in eight compass sectors (%)								
	E	SE	S	SW	W	NW	N	NE	P
0	33.11±3.87^c^	56.81±2.07^b^	52.65±2.26^b^	72.56±2.09^a^	65.13±0.43^a^	51.52±0.76^b^	31.74±4.59^c^	22.40±2.23^d^	0.000***
1	19.56±1.72^cd^	32.68±4.75^b^	32.89±1.11^b^	53.12±0.71^a^	46.71±0.65^a^	29.37±4.70^b^	25.32±2.28^bc^	13.70±1.18^d^	0.000***
2	11.56±2.50^d^	20.93±0.51^bc^	25.07±1.10^b^	41.16±3.08^a^	38.47±2.66^a^	25.75±4.18^b^	16.12±0.94^cd^	11.32±1.10^d^	0.000***
5	6.36±3.19^b^	11.25±1.23^b^	16.67±0.66^a^	22.00±1.80^a^	19.10±1.58^a^	9.83±1.41^b^	7.69±1.86^b^	4.70±0.43^b^	0.000***
10	6.67±3.33	6.41±0.26	6.56±0.87	13.03±2.65	8.15±0.94	4.76±4.76	3.90±1.98	1.45±1.45	0.137 NS
20	0	2.78±2.78	4.64±0.65	6.53±0.90	8.10±4.23	2.08±2.08	2.30±2.30	1.45±1.45	0.223 NS
30	1.67±1.67	0	1.08±1.08	2.56±2.56	2.22±2.22	1.85±1.85	0	1.15±1.15	0.913 NS
50	0	2.56±2.56	0	0	1.67±1.67	0	0	0	0.550 NS

Data are expressed as the average frequency of transgene flow at each distance and numbers in parentheses indicate the standard errors of the means. Different letters following the average values denote their significant differences (*P* < 0.05) under statistical analysis using the Student–Newman–Keuls (SNK) test. NS, not significant. ***P < 0.001.

Gene flow frequency in wheat followed an exponential decline as the distance increased in the eight compass sectors (Fig 3). Regression analyses were conducted for each direction and the results showed a high determination coefficient (R^2^) ranging from 0.851 to 0.968 (P<0.001), indicating that the exponential decay fitted well to the data and that the degree of simulation was relatively high (Table 2). The maximal frequencies of gene flow y at 60m and 80 m were 0.013% and 0.0002%, respectively, according to the simulation model *y* = 69.05 ∙ *exp*^(−0.22*x*)^ (R^2^ = 0.968). The exponential decay curve models for eight compass sectors revealed that there was a significant difference in the descending rate among the different directions and that the descending rate of curves in the higher frequency direction was relatively slow (Fig 3). An average transgene flow frequency of 48.24% in all compass directions was observed at 0 m distance from the pollen source. The frequency of transgene flow was reduced to 50% (O_50_) and 95% (O_95_) between 1.61 to 3.15 m, and 10.71 to 20.93 m, respectively.

**Fig 3:** Estimated regression curves showing the decrease of transgene flow frequencies from genetically modified (GM) wheat lines to dwarf male-sterile wheat (DMSW) with the increasing distance from the pollen source in eight compass sectors.

## Discussion

### Influence of wind direction on pollen and gene flow of transgenic wheat

Wheat is a self-pollinated crop with occasional outcrossing by wind-vectored pollen.

The likelihood and extent of pollen dispersal for wheat are considerably affected by meteorological factors, especially microclimatic conditions during the flowering period, such as wind speed and direction, ambient temperature and relative air humidity [7, 13, 29]. In this study, the average daily temperature was 21.6°C (with a mean of maximum temperatures of 24.3°C and minimum temperatures of 18.8°C) during the wheat flowering period, and the relative humidity was 63% (with a mean of maximum humidity of 78% and minimum humidity of 42%). The prevailing wind direction was ENE and E with the highest frequency in the flowering period. The average wind speed ranged from 1.2 to 3.3 m/s and the maximal wind speed was 2.8 to 5.9 m/s (Table 5). Our results indicated that the pollen flow of wheat differed significantly among the eight compass sectors, with higher pollen densities in the SW and W sectors, which were downwind and lower pollen densities in the NE, E, and N sectors, located upwind. Because the measurement of pollen flow was carried out on sunny days with calm atmospheric conditions in this study, wind direction may play a major role in wheat pollen dispersal under relatively stable microclimatic conditions.

**Table 5:** Meteorological data recorded during the wheat flowering period.

	Average	Relative	Prevailing	Maximum	Minimum	Average
	temperature (°C)	humidity (%)	wind direction	wind speed (m/s)	wind speed (m/s)	wind speed (m/s)
April 27	22.2	42	SSW	3.9	0.7	2.3
April 28	23.1	59	ESE	3.7	0	1.2
April 29	22.1	65	ENE	5.9	0.2	2.1
April 30	19	78	E	5.6	1.4	3.3
May 1	18.8	72	E	4.5	0.8	2.5
May 2	21.8	67	NW	3.8	1	2
May 3	24.3	57	ENE	2.8	0	1.2

Moreover, we found that the patterns of seed set and pollen-mediated gene flow were similar to that of pollen dispersal. The higher seed set and gene flow frequency sectors were detected in the same directions where we found more pollen grains, while the lower seed set and gene flow frequency sectors were detected in the directions with less pollen grain. These results are consistent with the findings of previous studies of pollen and gene flow in wheat, where different pollen density and gene flow frequency were observed in various directions. For example, with a 50 × 50 m pollinator block surrounded by recipient fields, the results showed that the elevated gene flow rates found to the N, W, and NW of the pollinator were closely associated with prevalent winds [11]. The field experiments were conducted using the blue aleurone wheat as pollen donor at five sites to determine the potential for pollen-mediated gene flow among winter wheat cultivars and found that the gene flow was generally in the direction of the prevailing wind and tended to occur more often at the sites where the sources were under lower temperature and higher humidity during pollination, suggesting that environmental factors had great impacts on the potential for pollen-mediated gene flow of wheat [16]. It is therefore necessary to conduct further detailed studies on the influences of weather parameters on the distribution of wheat pollen and gene flow under normal field conditions.

### The change of pollen and gene flow with increasing distance from pollen source

This study demonstrated that the density of transgenic wheat pollen decreased dramatically with the increase in distance from its source. Most of the pollen grains concentrated within 5 m and only a few pollen grains were detected at over 30 m. Seed setting of DMSW dropped sharply within short distance intervals, which indicated that the pollen donor transgenic wheat served as the main pollen source. Our results suggested that the seeds set of the pollen receptors and pollen-mediated gene flow were well correlated with the average pollen concentration at each distance. The frequency of transgene flow significantly declined with the deceasing pollen density from pollen source. Moreover, it is known that the lower gene flow frequency found at farther distances might be, to some extent, related to the reduction of pollen viability from the pollen donor [34, 35]. Previous studies found that the pollen of cultivated wheat loses 80% of its viability within 1 h of shedding from the anther at 20–25°C, temperatures commonly found during the wheat flowering period [21]. Thus, viable wheat pollen rarely travels long distances. Such findings further confirm that isolation distance should be a very effective method for minimizing crop-to-crop gene flow in wheat fields. This conclusion is remarkably consistent with the earlier studies on gene flow of wheat, which demonstrated that the transgene flow frequency or outcrossing rate was a function of distance and that isolation distance was the most effective method to regulate pollen-mediated gene flow for self-pollinating crops [16, 20]. However, in our study the maximal transgene flow frequency of 2.56% was detected at distance 50 m from pollen sources (Table 4), which was much higher compared to that reported in previous studies [22, 28]. This may be because DSMW without viable pollen was used as pollen receptor, while receptor variety was common wheat cultivar with low outcrossing rate in other studies.

### Relationship between Pollen competition and transgene flow frequency

In this study we used the DSMW as pollen receptor for two reasons: 1) to detect the gene flow of transgenic wheat in the absence of pollen competition; and 2) to easily investigate the effect of wind direction on gene flow frequency of transgenic wheat. Because the pollen receptors used in previous studies were usually common wheat cultivars, the gene flow frequencies of ~1% are relatively low [15, 28, 36]. It is difficult to distinguish the differences in gene flow frequency between the geographical orientations associated with the wind direction. In the present study, the allogamous DSMW does not produce viable pollen and, therefore, easily accepts foreign pollen [37, 38]. DSMW has a high rate of outcrossing and is thus an ideal material for the investigation of wheat gene flow or to amplify differences in gene flow frequency between geographical orientations, so as to reveal the association of gene flow with wind direction. In our experiment, we detected a maximal transgene flow frequency of 72.56% near the pollen source, while the mean frequency in all eight compass sectors was 15.95% (Table 4). It may be due to the different receptor variety, the gene flow frequency was much higher than that reported in other studies using common cultivar wheat, suggesting that the DMSW had a significantly amplifying effect.

It is worth noting that the maximal transgene flow frequency to the DMSW was 72.56% in this study, rather than the expected 100% if no pollen competition from non-transgenic plants was provided. This could be accounted for by non-dwarfing fertile plants being included as competitors around the DMSW receivers. Although we removed non-dwarfing plants by hand during the wheat flowering period, it is impossible to entirely remove all non-dwarfing plants from the DMSW populations. Consequently, non-GM pollen grains from fertile plants in air currents would compete with GM pollen grains from the pollen source, and the proportion of non-GM pollen grains relative to GM pollen was expected to increase with increasing distance from the pollen donor, which allowed the pollen of non-GM plants growing nearby the DMSW to be more easily received. A study reported that the frequency of PMGF from a herbicide-resistant (HR) volunteer population to a non-HR crop decreased exponentially with increasing plant population density of the crop because of pollen competition from the conventional wheat [35]. It should be pointed out that when there is no pollen competition and the experimental plot is strictly isolated, then the transgene flow frequency to the male sterile line could be estimated directly on the basis of the seed-setting rate.

## Conclusion

This study showed that pollen density and gene flow frequency of transgenic wheat were significantly different at various directions, suggesting that wind direction had a strong influence on the pollen dispersal and pollen-mediated gene flow of wheat. Pollen and gene flow frequency decreased sharply with increasing distance from pollen source and the descending rate was relatively slow in the prevailing or sub-dominant downwind directions. Our study confirmed that isolation by distance could effectively confine pollen from transgenic wheat and decrease the influence of pollen dispersal on seed purity. The density of GM pollen grains in air currents relative to the density of local non-GM pollen is important for transgene flow frequency, suggesting that further studies should investigate the impact of pollen competition (including internal and external) on transgene flow frequency. In addition, further impact factors, such as the outcrossing ability of the recipient, pollinator source size, wheat variety and other meteorological factors, should be studied in detail under different field conditions so as to determine the proper isolation distance and apply relevant agricultural production.

## Supporting Information

S1 Table Pollen density detected in eight compass sectors at different distance from pollen source. (DOCX)

S2 Table Transgene flow frequency detected in eight compass sectors at different distance from pollen source. (DOCX)
